# Clinical Application of Perioperative Anaesthesia Management Based on Enhanced Recovery after Surgery Concept to Elderly Patients Undergoing Total Knee Replacement

**DOI:** 10.1155/2022/8039358

**Published:** 2022-03-29

**Authors:** Jizheng Zhang, Jinli Che, Xiaohua Sun, Wanlu Ren

**Affiliations:** Department of Anesthesiology, Outpatient and Emergency,Tianjin Hospital, Tianjin 300211, China

## Abstract

**Objective:**

To explore the clinical application effect of perioperative anesthesia management based on enhanced recovery after surgery (ERAS) concept to elderly patients undergoing total knee replacement (TKR).

**Methods:**

By means of retrospective analysis, the medical data of elderly patients undergoing TKR treated in our hospital (02, 2019–02, 2020) were analyzed, and 100 patients were selected as the study objects according to the inclusion and exclusion criteria and divided into the study group (SG) and reference group (RG) according to their admission order, with 50 cases each. Patients in SG received perioperative anesthesia management based on ERAS concept, and those in RG accepted routine perioperative anesthesia management, so as to compare the perioperative inflammatory factors levels, postoperative recovery indicators, and postoperative Numeric Rating Scale (NRS) scores between the two groups.

**Results:**

Compared with RG after surgery, SG obtained significantly lower inflammatory factors levels (*P* < 0.001) and significantly better recovery indicators (*P* < 0.05), and the pain scores at postoperative 12 h and 24 h of SG were, respectively (1.46 ± 0.67) points and (2.00 ± 0.45) points, which were significantly lower than those of RG (*P* < 0.05).

**Conclusion:**

Perioperative anesthesia management based on EARS concept can improve the perioperative indicators of elderly patients undergoing TKR, result in less postoperative pain, and obtain a more desirable recovery.

## 1. Introduction

The knee joint is the main joint bearing weight on the lower extremities and is constituted by the lower femur, upper tibia, and patella, which is complex in structure and function, so the incidence of lesions remains high [1]. The incidence of knee joint diseases has increased significantly in recent years with rising aging globally, and survey data have shown that the aged population over 60 years old has a probability of developing knee osteoarthritis (OA) of more than 50.0%, while the aged population over 70 years old can have a prevalence of up to 70.0% [2], and the demand of total knee replacement (TKR) for elderly patients is elevating to improve their quality of life (QOL). As the primary treatment for end-stage knee OA, TKR can effectively relieve knee pain and improve patients' knee function, hence its clinical application is wider [3]. However, patients undergoing knee replacement are prone to postoperative complications such as pain, deep vein thrombosis, and pulmonary infection, in particular, the elderly patients with comorbid basic diseases such as diabetes mellitus and hypertension tend to have abnormal blood glucose index and blood pressure index, leading to higher complication rates [4, 5] and resulting in significantly increased length of hospital stay and hospital costs. To improve the surgical outcomes of elderly patients, current clinical efforts have been devoted to promoting the concept of enhanced recovery after surgery (ERAS), which refers to a multidisciplinary approach in the perioperative period to scientifically and effectively reduce the perioperative stress response and complication rate, thus reducing the incidence of infectious complications and chronic complications and achieving the goal of rapid rehabilitation [6, 7]. At present, ERAS concept has been mostly used in gastrointestinal surgery and urinary surgery [8], and most studies only focused on the effect of ERAS concept on patients' surgical indicators and QOL, and lacked the exploration of the central role of ERAS, i.e., reducing stress levels. The 2018 Anaesthesia Conference emphasized that the stress level, inflammatory reactions, and pain are the three essential elements in the perioperative period, moderate elements help to maintain a stable circulation, while excessive elements will increase the incidence of postoperative complications in patients [9, 10]. Anaesthesia is one of the most important factors in determining the levels of these elements, and scientific anaesthetic management can accelerate patient recovery by affecting the levels. Therefore, the study applied ERAS concept in perioperative anesthesia management for patients undergoing TKR, aiming to explore whether patients' postoperative recovery can be improved by standardizing anesthesia management with ERAS concept.

## 2. Materials and Methods

### 2.1. Study Design

It was a retrospective study conducted in our hospital (02, 2019–02, 2020) to explore the clinical application effect of perioperative anesthesia management based on ERAS concept on elderly patients undergoing TKR.

### 2.2. Enrollment of Study Objects

Inclusion criteria. (1) The patients were diagnosed with knee OA and met the indications of TKR [11]; (2) the patients were treated in our hospital in the whole course; (3) the patients had complete perioperative key data; (4) the patients did not have history of knee surgery; (5) the patients had normal deep veins of lower limb in the color ultrasound; (6) the patients used posterior stabilized cemented fixation; (7) the patients' anesthesia grade was II or III; and (8) the patients were at least 60 years old.

Exclusion criteria. (1) The patients' perioperative key data went missing; (2) the patients had diseases that might affect the study results; (3) the patients had mental disorder and could not communicate with others; and (4) the patients received bilateral knee replacement.

### 2.3. General Data of Study Objects

According to the inclusion and exclusion criteria, 100 patients were selected as the study objects and divided into the study group (SG) and reference group (RG) according to their admission order, with 50 cases each. In SG, there were 25 males and 25 females, with mean age of (72.48 ± 6.68) years, mean height of (160.10 ± 10.22) cm, mean body mass of (54.98 ± 4.65) kg, and mean BMI of (21.22 ± 1.23) kg/m^2^; before surgery, the numbers of patients complicated with hypertension and diabetes mellitus were respectively 20 and 18; there were 22 patients with grade II anesthesia, and 22 patients with grade III anesthesia; 29 patients received left knee replacement, and 21 patients received right knee replacement; in RG, there were 23 males and 27 females, with mean age of (72.36 ± 6.72) years, mean height of (160.23 ± 10.35) cm, mean body mass of (55.05 ± 4.21) kg, and mean BMI of (21.18 ± 1.22) kg/m^2^; before surgery, the numbers of patients complicated with hypertension and diabetes mellitus were respectively 22 and 20; there were 28 patients with grade II anesthesia, and 22 patients with grade III anesthesia; 27 patients received left knee replacement, and 23 patients received right knee replacement; No statistical between-group differences in general data including their age, height, body mass, anesthesia grade and replaced side were observed (*P* > 0.05), presenting comparability.

### 2.4. Moral Consideration

The study met the principles in the *World Medical Association Declaration of Helsinki (2013)* [12], and was approved by the ethics committee of *Tianjin Hospital*. After enrollment, the study team explained the study purpose, meaning, contents and confidentiality to the patients and asked the patients to sign the informed consent.

### 2.5. Methods

Patients in SG received perioperative anesthesia management based on ERAS concept, and those in RG accepted routine perioperative anesthesia management.

#### 2.5.1. Preoperative Assessment

Patients in SG were informed of the ERAS strategy before surgery by the anesthesiologist and were uniformly evaluated, and for those with hypertension and diabetes, blood glucose and blood pressure control was performed to improve preload and afterload and perioperative electrolyte balance, and the use of hypotensive drugs and hypoglycemic drugs in the perioperative period was adjusted. If patients were diagnosed with anemia before surgery, correction of hemoglobin to normal levels was required to reduce the rate of allogeneic blood transfusion and hospitalization costs. In addition, malnourished patients were assessed to determine whether they were at high risk, accepted 5–7 d of oral nutritional supplementation, and could drink clear fluids 2 h before surgery. Routine conversation was performed to patients in RG, informing the patients of the anesthesia modality and risks of TKR, and fasting and water deprivation management was conducted.

Before anesthesia, patients in SG were administered with ondansetron (manufactured: Sinopharm YiXin Pharmaceutical Co., Ltd.; NMPA approval no. H20053855) to prevent postoperative nausea and vomiting (PONV), and nonopioid analgesics and opioid analgesics were combined to improve the analgesic effect and suppress central sensitization. According to patients' preoperative evaluation, patients could selectively apply corticosteroid hormone, antacid drugs, etc., and attention was paid to the dosage applied to avoid postoprerative delirium. No intervention was performed to patients in RG.

#### 2.5.2. Intraoperative Anaesthesia

After entering the operating room, data of various vital signs were under routine monitoring, and the room temperature was maintained at 24–26°C. The selection of intraoperative anesthesia measures depended on factors such as anticoagulation state, cardiopulmonary state, and patients' intention, which mainly included general anesthesia and intrathecal anesthesia, and the later one was preferred in case of no related contraindications. According to patients' actual condition, tranexamic acid (manufactured: Shanxi Pude Pharmaceutical Co., Ltd.; NMPA approval no. H14020886) was selectively applied to reduce blood loss. The anesthesia maintenance scheme for SG was adjusted as required by intraoperative electrophysiologic monitoring, and under the circumstance of satisfying the need for surgical operation stimulus intensity, excessive intraoperative sedation should be avoided to reduce the possibility of postoperative delirium and cognitive impairment. Meanwhile, changes in blood pressure of patients in SG was under close monitoring, especially those with hypertension history, the arterial blood pressure was strictly controlled, and individualized blood pressure regulation objective was established. During surgery, heating with temperature-adjusting blanket and infusion heater was performed to patients in RG to make sure that their body temperature was maintained at over 36°C, and body monitoring was not performed. In addition, importance should be attached to intraoperative body fluid management and PONV prevention for both RG and SG. With either goal-directed or restrictive infusion, euvolemia and hemodynamic stability should be maintained for both groups to avoid volume overload or tissue edema. During surgery, dexamethasone (manufactured: Shanghai Andu Pharmaceutical Co., Ltd.; NMPA approval no. H20073181) could be administered to patients to prevent PONV, but it should be selectively applied to patients with diabetes.

#### 2.5.3. Postoperative Pain Management

Multi-mode postoperative analgesia scheme was performed to patients in SG, mainly the combined application of measures such as local infiltration anesthesia around the site undergoing knee replacement, and the drug used included local anaesthetic, opioids, non-steroidal anti-inflammatory drugs, and N-methyl-D-aspartate receptor antagonist. For patients in RG, routine analgesia measures were performed according to the actual situation.

### 2.6. Observation Criteria

1. Perioperative inflammatory factors levels. Before surgery, and 12 h and 24 h after surgery, 5 ml of peripheral venous blood was drawn from patients to centrifuge under 3,200 r/min for 10 min and then let stand for 30 min to extract the supernatant, and the levels of interleukin-6 (IL-6), interleukin-10 (IL-10), c-reactive protein (CRP) and tumor necrosis factor-*α* (TNF-*α*) were measured with enzyme linked immunosorbent assay (ELISA) (Beijing Kewei Clinical Diagnostic Reagent Inc.; NMPA approval no. S20060028).
2. Postoperative recovery indicators. ① Time of first off-bed activity and hospital stay after surgery of patients in the two groups were recorded; ② the occurrence of postoperative complications of patients were recorded; ③ patients' knee motion range and quadriceps muscle strength 7 days and 24 days after surgery were recorded.
3. Numeric Rating Scale (NRS). NRS score [13] was a pain scale suitable for elderly patients, which indicated the degree of pain with numbers 1–10, to be specific, a straight line was equally divided into 10 segments to indicate the degree of pain on a scale of 0–10 points, and patients drew circle on the numbers, with higher scores indicating stronger pain, and 10 points indicating severe pain keeping them awake. The NRS scores of patients before surgery, and 12 h and 24 h after surgery were recorded.

### 2.7. Statistical Processing

In this study, the data processing software was SPSS20.0, the picture drawing software was GraphPad Prism 7 (GraphPad Software, San Diego, USA), the items included were enumeration data and measurement data, the methods used were X^2^ test and *t*-test, and differences were considered statistically significant at *P* < 0.05.

## 3. Results

### 3.1. Comparison of Patients' Perioperative Inflammatory Factors Levels

After surgery, the inflammatory factors levels were significantly lower in SG than in RG (*P* < 0.001). See Figure 1.

### 3.2. Comparison of Patients' Postoperative Recovery Indicators

The postoperative recovery indicators were significantly better in SG than in RG (*P* < 0.05). See Table 1.

### 3.3. Comparison of Patients' Postoperative Pain Scores

After surgery, the postoperative 12 h and 24 h pain scores of SG were respectively (1.46 ± 0.67) points and (2.00 ± 0.45) points, which were significantly lower than those of RG (*P* < 0.05). See Table 2.

## 4. Discussion

ERAS concept refers to the implementation of various proved effective methods in the perioperative period, guided by evidence-based medicine, to reduce the intraoperative stress of patients and reduce the likelihood of postoperative complications, thereby improving their physical and mental status and accelerating the recovery process [14, 15]. Since it helps to reduce the perioperative mortality of patients, it is often applied in practice in the perioperative management of various types of malignancies, with common measures mainly including preoperative education, intraoperative management, intraoperative heat retention, and deep vein thrombosis prevention, of which anesthesia management belongs to one of the branches most significantly affecting the stress level of patients [16]. The stress response triggered by anesthesia causes a range of physiopathological changes in patients, including neurological, endocrine, metabolic changes, with important implications for patient outcome and prognosis [17]. Previous studies have suggested that the surgical stimulation resulting from anesthesia exerts a protective effect mainly by secreting hormones such as catecholamines through the hypothalamic-pituitary-adrenal axis and the sympathetico-adrenomedullary system and leading to stress response in the body. However, the sympathetic nerves are always chronically activated in older patients, whose neural tone is elevated, so they are highly susceptible to excessive stress reactions, which trigger a series of negative effects that lead to a systemic inflammatory response syndrome [18]. Elderly patients undergoing TKR have low surgical tolerance, tracheal intubation, postural changes, and expansion of medullary cavity all trigger hemodynamic fluctuations, so they often experience coughing and agitation during extubation, and their oxygen consumption is higher than that of other age groups, and in particular, those with comorbid cardio cerebrovascular diseases are more likely to experience severe cardio cerebrovascular and airway complications postoperatively [19]. Therefore, the regulated anesthesia management of elderly patients undergoing TKR based on ERAS concept can reduce their stress levels and improve their perioperative indicators.

Patients in SG were given preoperative health preaching and individualized assessment by anesthesiologists, which is beneficial to alleviate their anxiety and improve the perioperative cooperation. Patients with hypertension and diabetes must receive blood pressure and glucose control before operation, and can drink some water to improve circulation stability and reduce postoperative insulin resistance, thus accelerating the recovery of gastrointestinal function [20]. Ishii Yoshinori et al. showed that insulin resistance could be reduced if patients undergoing TKR were to eat and drink water moderately before surgery, and their hospital stay could be shortened to (8.54 ± 0.54) d [21], which was consistent with the results obtained herein. Not only that, the combination of preoperative analgesia and postoperative multi-mode analgesia can enhance the analgesic effect and alleviate central sensitization in patients. Leppänen Sanni et al. reported that multi-mode analgesia can reduce opioid use and alleviate adverse effects induced by analgesics, and that patients obtain more desirable analgesia effect, which is beneficial for enhancing their clinical satisfaction [22]. This study found that patients in SG had lower postoperative pain scores due to the multiple analgesic measures applied, which played a positive effect with small dose and high efficacy. Intraoperative anaesthetic measures and anaesthetic drugs did not differ between the two groups, but the amount of anaesthetic used by patients in SG was strictly controlled in an effort to avoid overuse of anaesthetic drugs when they met the stimulus intensity needs of the surgical procedure. In general, patients in SG received better measures of intraoperative heat retention and sedation, so they had less severe stress reactions, lower levels of inflammatory factors, reduced postoperative complication, and faster postoperative rehabilitation. It should be noted that no statistical analysis was performed on the incidence of postoperative cognitive impairment in the two groups in this study, but previous literature has shown that patients receiving quality anesthesia management are less likely to develop postoperative cognitive impairment [23–25], and the positive effect of ERAS concept in perioperative anesthesia management of elderly patients should be further explored in practice.

To sum up, perioperative anesthesia management based on EARS concept can improve the perioperative indicators of elderly patients undergoing TKR, result in less postoperative pain, and obtain a more desirable recovery. Promoting such perioperative anesthesia management is conducive to improving the prognosis of elderly patients and relieving medical burden.

## Figures and Tables

**Figure 1:** Comparison of patients' perioperative inflammatory factors levels (*x* ± *s*). *Note.* In the figure, the lines with dots indicated SG, and the lines with blocks indicated RG. (a) shows the IL-6 levels (pg/ml), which were not statistically different between SG and RG before surgery (5.65 ± 0.98 vs 5.67 ± 0.96), and were significantly lower in SG than in RG 12 h and 24 h after surgery (17.12 ± 2.65 vs 23.98 ± 2.65, 10.66 ± 0.98 vs 15.98 ± 1.50). (b) shows the IL-10 levels (pg/ml), which were not statistically different between SG and RG before surgery (5.44 ± 0.54 vs 5.42 ± 0.58), and were significantly lower in SG than in RG 12 h and 24 h after surgery (15.65 ± 2.65 vs 29.65 ± 2.68, 12.98 ± 1.65 vs 19.98 ± 2.65). (c) shows the CRP levels (mg/ml), which were not statistically different between SG and RG before surgery (25.44 ± 2.65 vs 25.50 ± 2.65), and were significantly lower in SG than in RG 12 h and 24 h after surgery (44.65 ± 2.63 vs 56.98 ± 4.65, 35.65 ± 2.41 vs 49.66 ± 2.41). (d) shows the TNF-*α* levels (ng/ml), which were not statistically different between SG and RG before surgery (18.65 ± 2.64 vs 18.74 ± 2.40), and were significantly lower in SG than in RG 12 h and 24 h after surgery (48.98 ± 2.65 vs 58.98 ± 2.65, 41.65 ± 2.65 vs 44.65 ± 2.58).

**Table 1:** Comparison of patients' postoperative recovery indicators.

Group	SG (*n* = 50)	RG (*n* = 50)	*X* ^2^/*t*	*P*
Time of first postoperative off-bed activity	6.74 ± 1.11	8.64 ± 1.10	8.597	<0.001
Postoperative hospital stay	8.11 ± 1.23	11.22 ± 1.54	11.158	<0.001
Complications				
Deep venous thrombosis	0 (0.0)	2 (4.0)	2.041	0.153
Dislocation of fixation	0 (0.0)	2 (4.0)	2.041	0.153
Pressure sore	1 (2.0)	3 (6.0)	1.042	0.307
Lung infection	2 (4.0)	4 (8.0)	0.709	0.400
Urinary tract infection	1 (2.0)	3 (6.0)	1.042	0.307
Complication rate	4 (8.0)	14 (28.0)	6.775	0.009
Knee motion range (°)				
Postoperative 7 d	78.65 ± 5.98	70.12 ± 4.65	7.962	<0.001
Postoperative 24 d	118.65 ± 8.10	112.65 ± 9.20	3.461	0.001
Quadriceps muscle strength (Nm)				
Postoperative 7 d	95.62 ± 1.65	92.65 ± 1.50	9.418	<0.001
Postoperative 24 d	110.65 ± 9.22	101.54 ± 9.65	4.827	<0.001

**Table 2:** Comparison of patients' postoperative pain scores (*x* ± *s*, points).

Group	SG (*n* = 50)	RG (*n* = 50)	t	*P*
Preoperative	4.56 ± 1.17	4.50 ± 1.25	0.248	0.805
Postoperative 12 h	1.46 ± 0.67	1.84 ± 0.76	2.652	0.009
Postoperative 24 h	2.00 ± 0.45	2.86 ± 0.75	6.953	<0.001

## Data Availability

Data to support the findings of this study is available on reasonable request from the corresponding author.
